The article "Rapid Dantrolene Administration with Body Temperature Monitoring Is Associated with Decreased Mortality in Japanese Malignant Hyperthermia Events" was published in 2023. Journal: Biomed Res Int.

# Rapid Dantrolene Administration with Body Temperature Monitoring Is Associated with Decreased Mortality in Japanese Malignant Hyperthermia Events

**DOI:** 10.1155/2023/8340209

**Published:** 2023-02-22

**Authors:** Yukari Toyota, Takashi Kondo, Daiki Shorin, Ayako Sumii, Kenshiro Kido, Tomoyuki Watanabe, Sachiko Otsuki, Rieko Kanzaki, Hirotsugu Miyoshi, Toshimichi Yasuda, Yousuke T. Horikawa, Keiko Mukaida, Yasuo M. Tsutsumi

**Affiliations:** ^1^Department of Anesthesiology and Critical Care, Hiroshima University Hospital, Hiroshima, Japan; ^2^Department of Anesthesiology, Hiroshima Prefectural Rehabilitation Center, Higashi, Hiroshima, Japan; ^3^Department of Pediatrics, Sharp Rees-Stealy Medical Group, San Diego, CA, USA

## Abstract

**Purpose:**

Malignant hyperthermia (MH) is a rare genetic disorder but one of the most severe complications of general anesthesia. The mortality rate of MH has dropped from 70% in the 1960s to 15% because of dantrolene, the only currently accepted specific treatment for MH. In this study, we retrospectively identified the optimal dantrolene administration conditions to reduce MH mortality further.

**Methods:**

Our database performed a retrospective analysis of patients with MH clinical grading scale (CGS) grade 5 (very likely) or 6 (almost certain) between 1995 and 2020. We examined whether dantrolene administration affected mortality and compared the clinical variables associated with improved prognosis. Furthermore, a multivariable logistic regression analysis was used to identify specific variables associated with improved prognosis.

**Results:**

128 patients met the inclusion criteria. 115 patients were administered dantrolene; 104 survived, and 11 died. The mortality rate of patients who were not administered dantrolene was 30.8%, which was significantly higher than those of patients who were administered dantrolene (*P* = 0.047). Among patients administered dantrolene, the interval from the first sign of MH to the start of dantrolene administration was significantly longer in the deceased than in the survivors (100 min vs. 45.0 min, *P* < 0.001), and the temperature at the start of dantrolene administration was also significantly higher in the deceased (41.6°C vs. 39.1°C, *P* < 0.001). There was no significant difference in the rate of increase in temperature between the two, but there was a substantial difference in the maximum temperature (*P* < 0.001). The multivariable analysis also showed that the patient's temperature at dantrolene administration and interval from the first MH sign to dantrolene administration was significantly associated with improved prognosis.

**Conclusions:**

Dantrolene should be given as rapidly as possible once MH has been diagnosed. Beginning treatment at a more normal body temperature can prevent critical elevations associated with a worse prognosis.

The article "Rapid Dantrolene Administration with Body Temperature Monitoring Is Associated with Decreased Mortality in Japanese Malignant Hyperthermia Events" was published in 2023. Journal: Biomed Res Int.

## 1. Introduction

Malignant hyperthermia (MH) is an autosomal dominant disorder that results in hypermetabolism of skeletal muscle. It is rare but one of the most severe complications of general anesthesia. The incidence of MH is 1-2 per 100,000 available anesthesia cases and higher in younger male patients, including neonates [1, 2].

Triggering drugs such as volatile anesthetics and depolarizing muscle relaxants increase the rate of Ca^2+^ release from the SR and exceed the speed of Ca^2+^ uptake by the SR, resulting in a sustained increase in intracellular Ca^2+^ concentration, resulting in uncontrollable skeletal muscle hypermetabolism. As a result, MH presents hypermetabolic reaction symptoms such as respiratory and metabolic acidosis, hyperthermia, muscular rigidity, fatal arrhythmia, and hypoxemia [3–5].

MH can be diagnosed clinically, which evaluates clinical presentation and laboratory findings, or MH can be diagnosed by *in vitro* testing, which examines the presence or absence of MH susceptibility, including a muscle biopsy and genetic analysis [6–8].

Although MH cannot be diagnosed by clinical presentation alone, identifying symptoms early is crucial to reduce mortality as MH can progress rapidly and become fatal. The clinical grading scale (CGS) is commonly used to assess the possibility of MH. The scoring system gives differential scores to the various clinical presentations of MH, and the scores are totaled to calculate the overall likelihood of MH [9]. Other criteria include Morio et al.'s clinical diagnostic criteria proposed in Japan, which emphasizes the importance of body temperature [10]. Despite these criteria, early diagnosis of MH has remained challenging because MH presents with variable hypermetabolic symptoms [11, 12]. Therefore, treatment should be initiated as soon as MH is suspected [1, 13].

In the 1960s, the mortality rate of MH in Japan was 70-80%. Since then, the mortality rate has decreased to about 15% due to the introduction of dantrolene [1]. However, today, the mortality rate remains at around 10% [1]. We hypothesized that the timing at which dantrolene was administered is essential to improve mortality and identified optimal conditions when to issue dantrolene.

## 2. Methods

### 2.1. Ethics

The retrospective cohort analysis was conducted by the principles of the Declaration of Helsinki, as revised in 2013. The study was approved by the ethics committee of Hiroshima University (Epidemiology-1081).

### 2.2. Data Collection and Patient Selection

Hiroshima University is a central MH research facility in Japan and is currently the only university that can perform the CICR test for a definitive diagnosis of MH. Our database of MH cases in Japan was created from anesthetic records, questionnaires, direct referrals from domestic facilities, and written case reports in domestic medical journals and conferences related to anesthesia. In addition, this database contains data from another institution, Saitama Medical University, that is used to perform the CICR tests. As a result, Hiroshima University has been collecting data on Japanese patients with MH since 1960, and our database reflects almost all of the MH cases in Japan [14].

The article "Rapid Dantrolene Administration with Body Temperature Monitoring Is Associated with Decreased Mortality in Japanese Malignant Hyperthermia Events" was published in 2023. Journal: Biomed Res Int.

We retrospectively investigated the MH CGS grade 5 (very likely) or grade 6 (almost certain) cases from our database that occurred between January 1, 1995, and December 31, 2020 (Figure 1). Patients that had insufficient data for analysis were excluded.

### 2.3. Retrospective Analysis of MH Cases

Patient demographics included patient age and sex. The frequency of succinylcholine and inhalant anesthetic administration was compared between survivors and deceased MH patients. The first signs suggestive of MH (first MH sign) were also compared in both groups.

The following recorded levels were collected: the frequency of dantrolene administration, timing of dantrolene administration, maximum rate of increase in body temperature, maximum body temperature, highest arterial partial pressure of carbon dioxide (PaCO_2_), highest end-tidal carbon dioxide (ETCO_2_), lowest arterial blood pH, lowest arterial base excess, highest creatinine kinase, highest serum myoglobin, and highest potassium. The rate of increase in temperature was evaluated over 15-minute intervals. Temperature abnormality was defined as a maximum temperature > 38.8°C or the rate of increase in temperature ≥ 0.5°C/15 min based on CGS and Morio's criteria [9, 10], respectively. We also compared the dose of dantrolene per body weight, body temperature at the start of dantrolene administration, and interval from the first MH sign to the beginning of dantrolene administration. In addition, the multivariate logistic regression analysis was performed with factors related to time and body temperature: body temperature at the start of dantrolene administration, maximum body temperature, the interval between anesthetic induction to first MH sign, and interval from the first MH sign to the beginning of dantrolene administration as explanatory variables and mortality as the objective variable, since previous reports have shown that maximum body temperature and early dantrolene administration are associated with MH mortality.

The article "Rapid Dantrolene Administration with Body Temperature Monitoring Is Associated with Decreased Mortality in Japanese Malignant Hyperthermia Events" was published in 2023. Journal: Biomed Res Int.

### 2.4. Statistical Analysis

Continuous variables were compared using the Mann–Whitney *U* test, and Fisher's exact test compared categorical variables. The logistic regression model calculated the adjusted odds ratio (OR) with a 95% confidence interval (CI). The findings were considered statistically significant when the *P* < 0.05. All statistical analyses were performed using Prism 8.0 software (GraphPad Software, San Diego, CA, USA).

## 3. Results

### 3.1. Patient Demographics and Characteristics

Our database has a total of 607 MH cases. 128 patients met the inclusion criteria, with 113 (88.3%) survivors and 15 (11.7%) deceased. There was no significant difference in the background characteristics between the survivors and the deceased (Table 1). The median age was 29 years (IQR, 15.0-52.0) for the survivors and 25 years (IQR, 11.0-53.0) for the deceased. Males were approximately 2.5 times more likely to experience an MH event.

### 3.2. First MH Sign

The most common first MH sign in all cases was elevated ETCO_2_ (55.8%), followed by temperature abnormality (19.5%) and sinus tachycardia (11.5%). However, among the deceased, sinus tachycardia was more common than temperature abnormality (Table 2).

### 3.3. Dantrolene Administration and MH Mortality

115 (89.8%) MH patients were administrated dantrolene, and 13 were not (Table 3). The mortality rate of patients not administered dantrolene was 30.8%, whereas that of patients given dantrolene was 9.6% (*P* < 0.047). The years and number of the fatal cases are listed as follows: 1 in 1995, 2 in 1996, 1 in 1997, 1 in 1998, 2 in 1999, 1 in 2001, 3 in 2002, 1 in 2006, 2 in 2008, and 1 in 2012.

### 3.4. Clinical Presentation

Our analysis revealed multiple significant differences between MH mortality outcomes. Maximum body temperature, peak serum myoglobin, and peak potassium were significantly higher in the deceased than in survivors. The lowest arterial blood pH and base excess were substantially lower in the deceased. The maximum rate of increase in temperature, maximum PaCO_2_, and maximum ETCO_2_ was not significantly different (Table 4).

### 3.5. Dantrolene Administration

There were no differences in the total dantrolene dose per body weight and the time interval from anesthetic induction to first MH sign between the survivors and the deceased (data not shown). The time interval from the first MH sign to dantrolene administration was significantly shorter in the survivors compared to the deceased (45 min (IQR, 25.0-75.0) vs. 100 min (IQR, 75.0-135.0), *P* = 0.007). The temperature at the start of dantrolene administration was significantly lower in the survivors (39.1°C (IQR, 38.6-40.3) vs. 41.6°C (IQR, 39.9-42.8), *P* < 0.001, respectively).

The article "Rapid Dantrolene Administration with Body Temperature Monitoring Is Associated with Decreased Mortality in Japanese Malignant Hyperthermia Events" was published in 2023. Journal: Biomed Res Int.

A logistic regression analysis was performed with the following four variables as explanatory variables and mortality as the objective variable: the time interval from anesthetic induction to first MH sign, maximum temperature, the temperature at dantrolene administration, and interval from first MH sign to dantrolene administration. The results showed that the body temperature at dantrolene administration and interval from first MH sign to dantrolene administration had a significant association with mortality (Table 5, *P* = 0.04 and 0.04, respectively).

## 4. Discussion

As previously reported, our study showed dantrolene's effectiveness in treating MH [15–17]. However, we also identified that a lower body temperature at the start of dantrolene administration and a shorter interval between the first MH sign and dantrolene administration were essential to reduce mortality.

Previous studies reported that the most common first MH signs were elevated ETCO_2_, sinus tachycardia, and masseter muscle rigidity [18, 19]. In our research, the most common first MH sign was elevated ETCO_2_, followed by temperature abnormality and tachycardia. Contrary to previous reports, in our patient population, temperature abnormality was observed in 94.5% of cases over the entire course, and in 19.5% was also the first sign of MH. Previous investigators have reported that temperature abnormality was only observed in approximately 86% of cases over the entire course of MH and only in about 8% of cases as a first sign [18, 19]. The North American Malignant Hyperthermia Registry of the Malignant Hyperthermia Association of the United States reported that without temperature monitoring, the mortality risk was 14 times higher, and the mortality rate was 30% [20]. The Japanese Society of Anesthesiologists (JSA) guideline for managing the MH crisis in 2016 states that continuous monitoring of ETCO_2_ and core temperature is essential in general anesthesia [1]. The advantage of temperature monitoring is that once the sensor is attached and measurement is started, changes over time can be observed continuously in a simple and noninvasive manner. Our results indicate that temperature monitoring should be started as early as possible while using anesthesia to identify any changes in body temperature which may suggest MH.

In an analysis of clinical characteristics during the entire course of MH events, maximum body temperature, serum and urine myoglobin, and potassium were significantly higher in the deceased than in the survivors, and arterial blood pH and base excess (BE) were substantially lower in the deceased. Although poor outcomes have been associated with metabolic acidosis and low BE in patients admitted to the intensive care unit, it remains unknown whether correction of metabolic acidosis improves prognosis in MH patients [21, 22].

The article "Rapid Dantrolene Administration with Body Temperature Monitoring Is Associated with Decreased Mortality in Japanese Malignant Hyperthermia Events" was published in 2023. Journal: Biomed Res Int.

Interestingly, there were no significant differences in the rate of increase in temperature, maximum PaCO_2_, or maximum ETCO_2_. The reason may be that the rise in ETCO_2_ is obscured by the increase in minute ventilation and therefore does not accurately reflect the progression of MH [23]. Reports from the North American Malignant Hyperthermia Registry (NAMHR) of the Malignant Hyperthermia Association (MHAUS) have also shown that ETCO_2_ cannot predict prognosis [20], and it has been recently reported that measurement of CO_2_ removal is necessary [24]. There was no difference in the dantrolene dose between the deceased and survivors, but the interval from the first MH sign to dantrolene administration was significantly longer in the deceased, and the temperature at the start of dantrolene administration was also significantly higher in the deceased.

The primary complications of MH include rhabdomyolysis, renal dysfunction, disturbance of consciousness, pulmonary edema, disseminated intravascular coagulation, and liver dysfunction, all of which may affect prognosis. Various studies have shown the relationship between MH complications and maximum temperature. It has been reported that a 2°C increase in maximum temperature is associated with a 2.9-fold increase in the risk of complications. That maximum temperature is an independent risk factor for complications, with higher temperatures associated with an increased risk of all complications [19]. In our study, the maximum temperature was approximately 2.0°C higher in the deceased than in the survivors, which may have affected the prognosis.

Recent studies have suggested that ryanodine receptor 1 (RYR1) plays an important role in heat-induced Ca^2+^ release and the progression to MH [25]. Furthermore, these data suggest a positive feedback mechanism altering thermogenesis causing MH. RYR1 mutant mice have been shown to have increased metabolic rates with increased Ca^2+^ leakage by volatile anesthetics [26, 27]. These data help suggest why temperature management early on is essential to MH mortality.

Dantrolene is the specific antidote for MH events. Early administration is associated with decreased complication risk and mortality [18, 20]. The univariate analysis limited to the cases administered dantrolene showed that the time from the first MH sign to dantrolene administration was longer in the deceased than in the survivors, and the maximum temperature and temperature at the start of dantrolene administration were higher. Multivariate analysis also showed that the temperature at dantrolene administration and interval from first MH sign to dantrolene administration was significantly associated with mortality. The European Malignant Hyperthermia Group (EMHG) guideline 2020 states that dantrolene should be available for administration within 5 min after recognizing the first MH sign [15]. There are also reports that the risk of complications increases 1.6-fold for every 30 min delay between the first MH sign and dantrolene administration and reaches 100% when the delay exceeds 50 min [18]. In Japan, a more soluble formulation of dantrolene (Ryanodex®, in 250 mg/vial to be reconstituted with 5 ml sterile water) has not been approved. Therefore, a less easily reconstituted dantrolene formulation, Dantrium (20 mg/vial after it is mixed with 60 ml of sterile water), must be used. If dantrolene is not immediately available, the temperature will continue to increase from when the prescription is requested until it is dissolved and administered. Our results suggest that monitoring temperature carefully after anesthesia induction and administering dantrolene expeditiously at a time when body temperature is less elevated may decrease MH event mortality.

The article "Rapid Dantrolene Administration with Body Temperature Monitoring Is Associated with Decreased Mortality in Japanese Malignant Hyperthermia Events" was published in 2023. Journal: Biomed Res Int.

Our study is limited as the database used in this study consisted of questionnaires and case reports from multiple institutions. As a result, missing data or a lack of uniformity in measurement criteria regarding clinical presentations may affect our interpretation of the results. We could not analyze the timing of blood collections as these were not known. Further accumulation of data is necessary for a more accurate understanding of the occurrence of MH in the future.

In conclusion, we investigated the clinical presentations and dantrolene administration in patients with MH in Japan since 1995. This study indicates the importance of quickly identifying MH and beginning dantrolene administration as crucial to improving prognosis. This will allow treatment to start at more normal body temperatures and prevent critical elevations associated with a worse prognosis. Developing protocols improving access to quickly obtaining and administrating dantrolene are essential to decreasing MH mortality.

## Figures and Tables

**Figure 1:** Patient selection criteria. MH: malignant hyperthermia; CGS: clinical grading scale.

**Table 1:** Characteristics of patients.

	Survivor (*n* = 113)	Deceased (*n* = 15)	*P* value
Age (yr), median (IQR)	29.0 (15.0-52.0)	25.0 (11.0-53.0)	0.54
Sex (male/female)	82/31	11/4	> 0.99
Body mass index, median (IQR)	21.6 (17.4-23.9)	22.5 (20.1-26.4)	0.27
Frequency of succinylcholine administration	24.3%	40.0%	0.22
Frequency of inhaled anesthetic administration	100%	100%	> 0.99

IQR: interquartile range.

The article "Rapid Dantrolene Administration with Body Temperature Monitoring Is Associated with Decreased Mortality in Japanese Malignant Hyperthermia Events" was published in 2023. Journal: Biomed Res Int.

**Table 2:** The first MH sign.

	Survivor (*n* = 113)	Deceased (*n* = 15)	Total
Temperature abnormality	19	3	22 (19.5%)
Elevation of ETCO_2_	57	6	63 (55.8%)
Sinus tachycardia	9	4	13 (11.5%)
MMR	10	1	11 (9.7%)
GMR	3	0	3 (2.7%)
Elevation of PaCO_2_	1	0	1 (0.9%)
Missing data	14	1	15 (11.7%)

Temperature abnormality was also defined as a maximum temperature > 38.8°C or rate of increase in temperature ≥ 0.5°C/15 min based on clinical grading scale and Morio's criteria [9, 10]. MH: malignant hyperthermia; ETCO_2_: end-tidal carbon dioxide; MMR: masseter muscle rigidity; GMR: generalized muscular rigidity; PaCO_2_: arterial partial pressure of carbon dioxide.

**Table 3:** Mortality differences according to dantrolene administration.

	Survivor (*n* = 113)	Deceased (*n* = 15)	Mortality (%)
Without dantrolene	9	4	30.8
With dantrolene	104	11	9.6

Odds ratio 0.24, 95% confidence interval 0.066-0.80, and *P* value 0.047.

**Table 4:** Clinical and biochemical presentations at dantrolene administration.

	Survivor (*n* = 104)			Deceased (*n* = 11)			*P* value
	Median	(IQR)	*n*	Median	(IQR)	*n*	
Maximum rate of increase in body temperature (°C/15 min)	0.80	(0.50-1.00)	93	0.65	(0.53-1.32)	8	0.81
Maximum body temperature (°C)	39.7	(38.8-40.9)	104	41.8	(39.9-43.0)	10	0.0017
Maximum PaCO_2_ (mmHg)	70.8	(56.4-89.0)	82	94.8	(48.7-152.1)	7	0.25
Maximum ETCO_2_ (mmHg)	75.0	(65.0-96.5)	81	84.0	(71.3-113.3)	4	0.45
Lowest arterial pH	7.17	(7.05-7.23)	82	6.96	(6.82-7.11)	8	0.0014
Lowest arterial base excess	-4.35	(−8.80-−2.00)	78	-14.05	(−19.9-−11.4)	8	< 0.0001
Highest creatinine kinase (IU/L)	3304	(1259-25766)	91	28064	(1723-223740)	8	0.12
Highest serum myoglobin (ng/mL)	1181	(659-1340)	35	24900	(1340-112000)	6	0.007
Highest potassium (mEq/L)	5.3	(4.5-6.0)	71	6.2	(5.0-7.6)	9	0.021
Dose of dantrolene (mg/kg)	1	(0.75-1.94)	27	0.98	(0.90-1.45)	7	0.70
Temperature at dantrolene administration (°C)	39.1	(38.5-40.3)	43	41.6	(39.9-42.8)	10	< 0.001
Anesthetic induction to first MH sign (min)	60.0	(30-130)	87	90.0	(15-165)	10	0.85
Interval from first MH sign to dantrolene administration (min)	45.0	(25.0-75.0)	43	100.0	(75.0-135.0)	5	0.007

Subjects with missing data were excluded. IQR: interquartile range; PaCO_2_: arterial partial pressure of carbon dioxide; ETCO_2_: end-tidal carbon dioxide; MH: malignant hyperthermia.

**Table 5:** Adjusted odds ratios of prognosis associated with the condition at dantrolene administration.

Explanatory variables	Odds ratio	95% CI	*P* value
Temperature at dantrolene administration (°C)	0.04	0.0009-0.57	0.04
Maximum body temperature (°C)	4.22	0.43-54.3	0.21
Interval from first MH sign to dantrolene administration (min)	0.96	0.92-0.99	0.04
Anesthetic induction to first MH sign (min)	1.01	0.99-1.02	0.46

MH: malignant hyperthermia; 95% CI: 95% confidence interval.

The article "Rapid Dantrolene Administration with Body Temperature Monitoring Is Associated with Decreased Mortality in Japanese Malignant Hyperthermia Events" was published in 2023. Journal: Biomed Res Int.

## Data Availability

Requests for data will be considered by the corresponding author.
